# Compressed Sensing Image Reconstruction of Ultrasound Image for Treatment of Early Traumatic Myositis Ossificans of Elbow Joint by Electroacupuncture

**DOI:** 10.1155/2021/4066415

**Published:** 2021-12-07

**Authors:** Yi Zhu, Mengyuan Sheng, Yuanming Ouyang, Lichang Zhong, Kun Liu, Tan Ge, Yaochi Wu

**Affiliations:** ^1^Department of Traumatology Acupuncture and Massage, Sixth People's Hospital Affiliated to Shanghai Jiaotong University, Shanghai 200233, China; ^2^Innovation Base Hospital of Jiangxi University of Traditional Chinese Medicine, Jiangxi, Nanchang 330004, China; ^3^Department of Orthopaedics, Sixth People's Hospital Affiliated to Shanghai Jiaotong University, Shanghai 200233, China; ^4^Department of Medical Ultrasonics, Sixth People's Hospital Affiliated to Shanghai Jiaotong University, Shanghai 200233, China; ^5^School of Information Engineering, Shanghai Maritime University, Shanghai 201204, China; ^6^Department of Preventive Medicine, Guangming Traditional Chinese Medicine Hospital, Shanghai 201399, China

## Abstract

This article conducts a retrospective analysis of 500 patients with posttraumatic elbow dysfunction admitted to our department from March 2019 to September 2020. The average time from injury to operation is 11 months (2–20 months). We adopt a personalized treatment method to completely remove the hyperplastic adhesion tissue and heterotopic ossification around the joint, remove part of the joint capsule and ligament, and release it to achieve maximum function. After the operation, an external fixator was used to stabilize the loosened elbow joint, and the patient was guided to perform rehabilitation exercises with the aid of a hinged external fixator, and celecoxib was used to prevent heterotopic ossification. Mayo functional scoring system was used to evaluate the curative effect before and after surgery. The rapid realization of ultrasound imaging under the framework of compressed sensing is studied. Under the premise of ensuring the quality of ultrasound imaging reconstruction, the theory of ultrasound imaging is improved, and a plane wave acoustic scattering ultrasound echo model is established. On this basis, the theory of compressed sensing is introduced, the mathematical model of compressed sensing reconstruction is established, and the fast iterative shrinkage thresholding algorithm (FISTA) of compressed sensing reconstruction is improved to reduce the computational complexity and the number of iterations. This article uses FISTA directly to reconstruct medical ultrasound images, and the reconstruction results are not ideal. Therefore, a simulation model of FISTA training and testing was established using the standard image library. By adding different intensities of noise to all images in the image library, the influence of noise intensity on the quality of FISTA reconstructed images is analyzed, and it is found that the FISTA model has requirements for the quality of the images to be reconstructed and the training set images. In this paper, Rob's blind deconvolution restoration algorithm is used to preprocess the original ultrasound image. The clarity of the texture details of the restored ultrasound image is significantly improved, and the image quality is improved, which meets the above requirements. This paper finally formed a reconstruction model suitable for ultrasound images. The reconstruction strategy verified by the ultrasound images provided by the Institute of Ultrasound Imaging of a medical university has achieved a significant improvement in the quality of ultrasound images.

## 1. Introduction

The elbow joint is a hinged upper limb joint composed of multiple joints such as the brachial ulnar joint, the brachioradial joint, and the upper radioulnar joint [1]. At the same time, an elbow joint with a good range of motion is very important for people's daily life and work. In order to meet the basic needs of people's daily work and life, our elbow joint needs to have at least 100° of flexion and extension range of motion, and at least 100° of forearm rotation range of motion. Among them, the minimum angle that the elbow joint can reach is less than 30°, the maximum angle that can be achieved by flexion is greater than 130°, and the angle of pronation and supination of the forearm needs to be greater than 50°. When the minimum extension angle of the elbow joint is greater than 30°, or the maximum flexion angle of the elbow joint is less than 120°, we define it as elbow joint stiffness. However, as one of the most important joints in the whole body, the elbow joint cannot tolerate the complications and sequelae caused by trauma [2]. Studies have shown that if the range of motion of the elbow joint is reduced by 50°, 80% of the elbow joint function will be lost [3]. With the rapid development of science and technology in today's society, more and more patients suffer from elbow joint trauma. The contracture of the soft tissue around the elbow joint caused by immobilization can cause the stiffness of the elbow joint after trauma [4].

In recent years, sparse signal processing technology has gained great attention in signal processing [5]. The establishment and rapid development of sparse signal processing theory, especially compressed sensing theory, has laid a theoretical basis for using sparse signal processing technology to solve actual signal processing problems. More and more applications are used to solve practical problems such as the slow speed of MRI data acquisition [6]. Compressed sensing, as a new sparse signal processing theory, provides us with a framework for sparse signal reconstruction using a small amount of measurement data. Based on this theory, we can greatly reduce the sampling data in the Fourier transform domain, shorten the data scanning time, and increase the imaging speed. This not only reduces the patient's discomfort during the scanning process but also enables the reconstruction of high-quality images from less Fourier data. Compressed sensing is a linear incomplete signal acquisition method, which mainly involves the sparsity of the signal, the acquisition of perceptual signals, and the reconstruction of perceptual signals. It breaks through the limitations of traditional sampling methods and opens a new era of sparse signal research. Many scholars are committed to this area of research, and a series of research results have appeared in just a few years [7, 8]. These studies mostly focus on the sparseness analysis of the signal, the design of the measurement matrix, the optimization of the reconstruction algorithm, and the practical application.

In this study, we collected the case data of 500 patients with posttraumatic elbow joint dysfunction after surgical treatment, revisited the recovery effect of elbow joint function, and explored the surgical treatment of posttraumatic elbow joint dysfunction. Surgical treatment of posttraumatic elbow joint dysfunction is the only option. Individualized treatment is used during the operation. A combined lateral and posterior medial incision is routinely used to completely remove the heterotopic bone tissue that blocks joint movement. This paper studies the compressed sensing theory and sparse reconstruction algorithm. First, the compressed sensing theory is explained, and then two reconstruction algorithms suitable for solving large-scale observation matrices are introduced: SPGL1 and FISTA. We reduce its computational complexity, speed up the convergence speed, and verify that the improved FISTA algorithm is still suitable for ultrasound imaging reconstruction. The relevant factors affecting the reconstruction of ultrasound images are studied, the training set image types and training set image quality are discussed, and the relevant sensitive variables are adjusted and improved on the basis of the FISTA network. After verification, the PSNR value of the ultrasound image reconstruction using FISTA is higher than other algorithms, which shows that FISTA has a certain effectiveness in ultrasound image reconstruction.

## 2. Related Work

For the diagnosis of fractures, plain radiographs, CT, and MRI have become more mature. The diagnostic value of ultrasound for fractures makes up for the shortcomings of plain radiographs, CT, and MRI in some aspects. Due to the flexibility and real-time characteristics of ultrasound, for some fractures with irregular bones or unclear displacements, the fracture can be diagnosed quickly by changing the position or angle of the probe, and it can also guide the fracture technique in time. In the case of complex trauma fractures, it can help determine whether there is substantial visceral damage, and the CDFI technology can be used to diagnose whether the blood vessel has combined damage. For fracture healing monitoring, CDFI can be combined to help evaluate and predict the causes of delayed fracture union and nonunion.

The use of high-frequency ultrasound combined with CDFI technology to examine soft tissue hemangioma reveals tortuous and expanded tubular structures that communicate with each other and interspersed with moderately strong echoes or strong echoes with sound shadows. Related scholars believe that CDFI can more accurately indicate the source of the main blood vessel supply and the scope of invasion of hemangioma, so as to provide a reliable basis for surgery, and it is low cost and noninvasive, with no X-ray injury [9]. Although the nature of other soft tissue tumors cannot be clarified by ultrasound, the appearance, internal echo structure, peripheral boundary conditions, blood flow conditions, and whether there is infiltration into surrounding structures can be preliminarily treated by ultrasound for benign and malignant tumors. Relevant scholars summarized 53 cases of soft tissue masses in other parts of the maxillofacial area except for maxillofacial area using CDFI technology [10]. All the bleeding flow velocity and resistance index were measured, and they found that there was a significant difference in the maximum blood flow velocity around benign and malignant tumors. Related scholars summarized the CDFI test results of 35 cases of soft tissue masses in the limbs and finally concluded that the arterial flow velocity of the malignant tumor group was significantly higher than that of the benign tumor group, and the resistance index was also significantly higher than that of the benign tumor, with Vs ≥ 015 m·s^−1^ as the demarcation standard for judging benign and malignant tumors [11].

Signal sparsity is a prerequisite for the application of CS theory. Almost all signals in nature are not sparse. The research on signal sparsity is a major difficulty in the application of CS theory. Related scholars have proposed a method of using contourlet transform as an image sparse transformation [12]. First, the image is decomposed into multiple detail subbands of different resolutions and a low-frequency subband, and then Hilbert transform is performed on the detail subbands. Finally, the two-dimensional analysis signal is decomposed by a directional filter bank, and the contourlet transform with translation invariance is realized. Experimental results show that contourlet transform has obvious advantages in image denoising and compressed sensing sparse signal [13]. Related scholars have proposed a method of using nonsubsampled contourlet transform as the sparse representation of the image in compressed sensing image reconstruction [14]. This method needs to measure the transformed high-frequency subbands and retain the decomposition coefficients of the low-frequency approximation subbands. The method not only improves the speed of image reconstruction but also guarantees the quality of image reconstruction. In addition, some scholars have used mixed sparse basis to sparse the signal, reduce the calculation time, and improve the accuracy of signal reconstruction. Related scholars have designed an orthogonal dictionary, which is composed of multiple orthogonal bases, which can adaptively find the optimal orthogonal base that approximates a certain signal characteristic and select the most suitable orthogonal base according to the different signals [15].

With the increasing role and use of high-frequency ultrasound in the diagnosis of muscular, skeletal, and neurological diseases, CDFI has gradually been found to have its inherent limitations. For example, when the gain is too high or the threshold is too low, the noise can easily cover the blood streaming signals, as well as the dependence on the angle and the proneness to aliasing. Under this circumstance, a new detection technology, namely, PDI, came into being. Its dynamic range improves the sensitivity to blood flow. The above advantages of PDI technology broaden the clinical application of CDFI, enabling accurate display of low-velocity blood flow and extremely low-velocity blood flow that were difficult to detect in the past, especially the detection of blood flow in small blood vessels, which significantly improves the sensitivity of doppler blood flow detection. However, PDI technology has its own shortcomings. For example, the application of PDI is limited for organs with obvious movement. PDI cannot display the direction and speed of blood flow, as well as direct quantitative values such as resistance index and maximum systolic peak, so it can only be used as a supplement to CDFI [16–18]. However, with the in-depth study of CDFI and PDI in musculoskeletal neurological diseases, it has shown good prospects [19, 20]. It is believed that high-frequency ultrasound will be an indispensable imaging method for the diagnosis of musculoskeletal neurological diseases in the near future.

## 3. Materials and Methods

### 3.1. General Information

From March 2019 to September 2020, patients who received elbow joint adhesion release in our hospital, a total of 500 patients with elbow joint dysfunction, were included, aged 10 to 64 years old, with an average age of 35 years. There are 300 cases on the left and 200 cases on the right joints. There were 280 cases of fall injuries and 220 cases of car accident injuries (all combined injuries). The average operation time was 11 months (2–20 months) after trauma. Original cause was as follows: 8 cases of simple elbow joint dislocation, 24 cases of humeral fractures, 8 cases of radial head fractures, 16 cases of olecranon fractures, 12 cases of horror triad, and 7 cases of multiple elbow fractures.

Education level was as follows: 50 cases in elementary school, 50 cases in junior high school, 100 cases in high school, and 300 cases in university; these patients all received surgical treatment for posttraumatic elbow joint dysfunction. Patients with posttraumatic elbow joint dysfunction were treated at 3 months, 6 months, and 12 months after surgery. Follow-up was done monthly and at 24-month time points, using the Internet (QQ or Email), telephone, and outpatient services to conduct a return visit to record the recovery of elbow joint function, elbow joint flexion and extension angle, rotation angle, joint pain, and stability. The enrollment followup time was all >6 months.

### 3.2. Treatment Methods

#### 3.2.1. Preoperative Preparation

We check the elbow joint flexion and extension range of motion, rotation range of motion, muscle strength, and neurological symptoms in detail and perform routine X-ray and CT plain scan + three-dimensional reconstruction before surgery to understand whether the articular surface is flat and whether the joint space is narrow and judge whether there is an ectopic position.

#### 3.2.2. Surgical Method

All patients in this group underwent surgical treatment after hospitalization. Brachial plexus block anesthesia was used in the operation, the affected limb was placed on the hand rest, sterile airbag tourniquet was used at the proximal upper arm after disinfection and drape, and the combined lateral and posterior elbow approach was routinely used. For patients with elbow joint dysfunction after one-stage surgical treatment, we use the original surgical incision and make a posterior medial or lateral incision at the same time; for patients with the original posterior median incision, we use the original posterior median single incision to take care of both the medial and the lateral sides; the medial incision exposes the ulnar nerve. We loosen the triceps brachii tendon, open the rear olecranon fossa, remove the fibrous scar tissue and granulation tissue, and remove the heterotopic ossified bone in the fossa; the lateral incision is from the brachioradialis muscle and extensor carpi radialis longus muscle, exposing the front joint capsule, coronal fossa, exposing the brachioradial joint, clearing the hypertrophic joint capsule and fibrous scar tissue, and heterotopic ossification of bone. Obstacles undergo resection of the radial head or replacement of the radial head prosthesis. Old fractures of the ulna coronoid process cannot be anatomically reduced and fixed. We routinely use nonabsorbable sutures to repair the anterior joint capsule to enhance the anterior stability of the elbow joint. The injured medial and lateral collateral ligaments are often separated and repaired. In this group of 500 patients, both the internal and external collateral ligaments were repaired. If necessary, Anchor rivet ligament stops were reconstructed and sutured. At the same time, the ulnar nerve is released before (or the medial condyle osteotomy is performed in situ) and placed under deep fascia for protection to avoid postoperative rehabilitation exercises and compression of the ulnar nerve. After the wound is fully hemostatic, a negative pressure drainage tube is placed in the incision; two external fixation nails are injected into the upper middle 1/3 of the humerus and the middle and lower 1/3 of the ulna (or distal radius), respectively, and the hinged external fixation is connected. The average operation time is 160 min (120–180 min).

#### 3.2.3. Postoperative Treatment

Routine use of dehydration drugs after surgery, local ice on the elbow that night, functional rehabilitation exercise under the guidance of a rehabilitation physician on the first day after surgery, active and passive functional exercises of the elbow joint with the aid of a hinged external fixator, and joint activities were performed. The scope depends on the patient's tolerance, and the elbow joint should not be moved under violence. Anti-inflammatory, swelling and pain relief oral celecoxib 200 mg/Bid prevents myositis ossificans. The drainage tube is placed for 10 to 12 days to fully drain the blood in the joint. The stitches were removed within 14 days, and the hinged external fixation bracket was removed for 6 to 8 weeks.  Figure 1 shows a schematic diagram of a specific exercise plan after elbow joint dysfunction release.

## 4. Ultrasonic Imaging Reconstruction Algorithm under the Framework of Compressed Sensing

### 4.1. Compressed Sensing

According to the signal theory, the signal can be expressed by a set of base linear, namely,

(1) $$\begin{array}{c} x=\sum_{n=0}^{N-1}a_{n}•\theta_{n}. \end{array}$$

In the formula, *a* is a coefficient vector of *N* ∗ 1. If there are only *K* nonzero coefficients (or coefficients far greater than zero) in the formula, then the signal *x* is said to be sparse (compressible) on the basis, and *θ*_*n*_ is called the sparse basis or sparse dictionary of the signal *x*, and *K* is the sparseness of the signal.

In the compressed sensing theory, the observation of the sparse signal *x* does not directly measure the signal *x* itself. Instead, the signal *x* is projected onto a set of low-dimensional measurement vectors through noncorrelated measurements, namely,

(2) $$\begin{array}{c} y=\eta x. \end{array}$$

In the formula, *y* is the vector of *M* ∗ 1, and *η* is the observation matrix of *M* ∗ *N*.

Since the signal measurement value dimension *M* is much smaller than the signal dimension *N*, directly solving the above equation is an underdetermined problem, and generally speaking, there is no definite solution. Considering the sparsity of a, this problem is expected to find a definite solution. The finite isometric property gives the necessary and sufficient conditions for the existence of a definite solution. To fully reconstruct the signal, it must be ensured that the observation matrix will not map two different *K*-item sparse signals to the same sampling set. This requires that the matrix composed of every *M* column vector extracted from the observation matrix is nonsingular. Practice has proved that most uniformly distributed random matrices have this condition, such as a matrix that obeys the Gaussian distribution, a matrix that obeys the Bernoulli distribution, and a part of the Fourier matrix.

### 4.2. Determine the Reconstruction Algorithm

In actual ultrasound imaging, the number of linear ultrasound array elements can be selected as 128. Assuming that the number of sampling points in the frequency domain is 64–128, considering the complex number, the size of the observation matrix *G* required for a detection area of 256 ∗ 256 pixels is 8–16 GB (storage in double-precision mode). It is undoubtedly huge. On the one hand, the computer's memory is required to support so much data. On the other hand, even if a solid state drive SSD is used to transfer data from the disk to the memory RAM at a speed of 500 MB/s, it will take 16–32 s, and the speed of an ordinary SATA3.0 hard drive will be reduced to the order of a minute.

As the amount of data increases, the processing time of data will also increase. According to the definition of algorithm complexity, the calculation time of the same algorithm will increase exponentially as the amount of data increases. Therefore, the calculation time after increasing the amount of data will far exceed an *O*(*N*2) complexity algorithm.

Therefore, in view of the characteristics of ultrasound imaging data, it is necessary to choose an algorithm that supports complex number operations, has lower algorithm complexity for large-scale matrices, and can converge as quickly as possible. We will focus on the SPGL1 algorithm and the FISTA algorithm. These two algorithms have a similar design basis, the gradient descent method, which belongs to the convex relaxation method in the reconstruction algorithm.

#### 4.2.1. SPGL1

It is mainly used to solve the BPDN (Basis Pursuit Denoising) problem. The BPDN problem is a variant of the BP problem. The expression is

(3) $$\begin{array}{c} \min{\left\|a\right\|}_{1}\;s.t.\;y-\sigma \leq a\theta . \end{array}$$

To solve the BPDN problem, the Least Absolute Shrinkage and Selection Operator (LASSO) problem is needed. The expression of the LASSO problem is

(4) $$\begin{array}{c} \min{\left\|a\theta -y\right\|}_{2}\;s.t.\;{\left\|a\right\|}_{1}\geq \tau \theta . \end{array}$$

From the perspective of expression, the LASSO problem is a dual representation of the BPDN problem; that is, the objective function of LASSO is the constraint condition of BPDN, and the constraint condition of LASSO is the objective function of BPDN.

Every iteration needs to judge whether it drops. If it does not, the iteration step size must be reduced until the descending condition is met; after the iteration is completed, the iteration step size needs to be updated with the help of the Barzilai-Borwein (BB) algorithm to ensure the overall situation. The core part of the SPG algorithm is gradient projection. From the classic gradient descent method, we can see that the update of a is determined by the following formula:

(5) $$\begin{array}{c} a_{k}=a_{k-1}+g•u•\eta , \end{array}$$

where *g* represents the gradient, *u* represents the iteration step size, and the gradient projection is to bring the right half of the above formula into the soft threshold iteration function *P*(), so that it satisfies

(6) $$\begin{array}{c} P\left(c\right)=\min{\left\|2a-c\right\|}_{2}\;s.t.\;{\left\|a\right\|}_{1}\geq \tau , \end{array}$$

where *c* represents the soft threshold. After the soft threshold processing, the elements in a that are smaller than the threshold will be set to 0, and the nonzero information will be concentrated in a few nonzero points, and the sparsity will slowly manifest.

#### 4.2.2. FISTA

It is an improved version of the iterative shrinkage threshold algorithm ISTA. The iterative shrinkage threshold algorithm is a very classic algorithm. It can solve the following regularization problems:

(7) $$\begin{array}{c} \min\left\{F\left(x\right)=\left[ay^{2}-\theta {\left\|\lambda a\right\|}_{2}\right]\right\}, \end{array}$$

where *λ* is called the regularization parameter.

The core of the ISTA algorithm is the gradient descent method, which is similar to SPGL1 in that it adds a threshold function *P*():

(8) $$\begin{array}{c} a_{k+1}=P_{\lambda u}\left[a_{k}-u\theta \left(y-ua_{k-1}\right)\right]. \end{array}$$

It can be a soft threshold or a hard threshold. This algorithm is very simple, but it has the same problems as the gradient descent method of slower convergence speed and uncertain global convergence. Therefore, what FISTA needs to do is to make the algorithm simple and fast convergent on the basis of ISTA, while ensuring global convergence. The flow of the FISTA algorithm is shown in Figure 2.

It can be seen from Figure 2 that the calculation process of FISTA is relatively simple, and there are three places that take time: one is to determine the iteration step size *u*; the other is to calculate the variable *z* when a matrix *θ* and a vector are multiplied. The variable *u*_*k*_ requires a conjugate transpose of the matrix *θ* and the vector multiplication operation, which is similar to SPGL1 in terms of computational complexity. But the process of FISTA is much simpler than that of SPGL1. SPGL1 needs to do outer loop and inner loop, and there are many branches at the same time. This may improve the robustness of the algorithm, but the reconstruction speed will be slower than FISTA.

### 4.3. FISTA Algorithm Optimization

#### 4.3.1. Optimization of Iteration Step Size

It can be seen in Matlab that if the SVD function is used to find the maximum singular value of the matrix, when the matrix dimension increases, the calculation time accounts for about 88%. From the perspective of algorithm time, it is the most time-consuming part. From the perspective of algorithm design, the iteration step size *u* taking the reciprocal of the largest singular value can ensure the fastest convergence speed, but it does not mean that the iteration step size is unique.

The optimization ideas for the iteration step size *u* are as follows: (1) open up a vector sum of length *N*; (2) add the absolute value of each column of the matrix *θ* and save it in sum[*i*]; (3) take sum of second norm, then take the reciprocal; this reciprocal is the estimated iteration step size *u*.

#### 4.3.2. Optimization of the Number of Iterations

In the experiments in this paper, the iteration number can meet the iteration requirement at 100 times. Since each iteration requires two matrix and vector multiplications, when the matrix dimension is relatively high, the time increases exponentially. After the iterative step size is optimized, the most time-consuming process in the FISTA algorithm is undoubtedly the iterative process, so it is necessary to optimize the iterative process.

Considering that the characteristic of ultrasound images is to find the nonuniform area in the detection area, that is, the exact location of the lesion is what we want to know most, as for the amplitude information of the nonuniform area, it is relatively less important and can be passed through the image. From this point of view, the number of iterations can be appropriately reduced. The function of the threshold function is to set the threshold so that the number below the threshold is set to 0, and the number above the threshold is subjected to threshold processing. Therefore, appropriately increasing the threshold will be an effective way to reduce the number of iterations.

Blindly increasing the threshold will cause the effective information to be set to 0, and the result will be inaccurate. Therefore, it is necessary to select an appropriate threshold to meet the needs of different scenarios. In this paper, based on the approximate normalization of the observation matrix, the value range of *λ* is defined as 2*e*^4^∼4*e*^4^, and 0.5*e*^4^ is used as a step size to adapt to different amounts of data to obtain the best reconstructed image effect and the threshold that reconstructs the least sparse point can finally reduce the number of iterations to 30. After the improvement, the time of each part of the FISTA algorithm is shown in Table 1.

## 5. Experiment and Analysis

### 5.1. The Impact of Training Set Image Types on Reconstruction Results

The experiment is divided into three groups: (1) the first group uses the 91-image library to train the FISTA network and then uses the trained network to perform superresolution reconstruction of the ultrasound images. (2) The second set of experiments uses Ultrasound Image Database to train the network. The database contains 84 ultrasound images from ten volunteers of different ages and weights. It is currently a common gallery in the field of ultrasound image research. (3) The third set of experiments uses the mixed training set of the previous two experiments to train the network. We compare the reconstruction effects of the trained network on ultrasound images in these three cases. Here is just to change the type of training set image, other experimental parameter settings, experimental schemes, etc. remain unchanged.

The experimental results are shown in Figures 3 and 4. Among them, US-FSRCNN1 represents a network trained using ultrasound images as a training set, FISTA represents a network trained using 91-image library as a training set, and FSRCNN represents a network trained using a mixed set.

It can be seen from Figures 3 and 4 that the PSNR and SSIM values of the ultrasound image reconstruction results obtained using the latter three methods based on compressed sensing are higher than those of the bicubic interpolation method. This shows that the ultrasound image reconstruction method based on compressed sensing is more effective than the general interpolation method. In addition, the network trained using ultrasound images as the training set has better reconstruction effects on ultrasound images than the network trained using the 91-image training set and the mixed training set. This fully proves that the network trained with a targeted training set has a better reconstruction effect on this type of image. Therefore, when training the network structure, a training set that is consistent with the type of image to be reconstructed should be used.

The comparison chart of the reconstruction results of ultrasound images is shown in Figure 5. From the visual point of view, we compare the reconstruction results of the four methods of bicubic interpolation, FSRCNN, US-FSRCNN1, and FISTA. We found that the first three methods have little difference in the reconstruction effect of ultrasound images. The network obtained by FISTA has the best reconstruction effect on ultrasound images. This verifies that the network trained with the FISTA ultrasound image training set can learn the characteristics of relevant ultrasound images in a targeted manner and is effective for ultrasound image reconstruction.

### 5.2. The Effect of Training Set Image Quality on the Results of Ultrasound Image Reconstruction

In the algorithm comparison experiment, this article adds speckle noise of different intensities to the 91-image training set to obtain multiple training sets of different qualities. By using these training sets to train the corresponding network, we discuss the impact of the training set under different intensities of noise on the effect of image reconstruction. The results show that FISTA has a certain antinoise ability.

When the added noise variance is greater than 0.04, the reconstruction effect of FISTA is already not ideal. At this time, the PSNR value of the training set is about 28.1237 dB. We conclude that, in order to get a better reconstruction effect, the image quality of the training set should be similar to the quality of the test image to be reconstructed.

FISTA is the best for ultrasound image reconstruction. Therefore, the following experimental results are compared with FISTA. The experimental results are shown in Figures 6 and 7. Among them, US-FSRCNN1 represents the network trained using the preprocessed training set. It can be seen from the figure that the reconstruction effect of the ultrasound image obtained by the network trained with the preprocessed training set is better than that of the nonpreprocessed training set. This verifies that the texture details of the training set images after preprocessing have been improved to meet the requirements, thereby improving the quality of the reconstructed image.

### 5.3. Comparison of Reconstruction Time with Other Algorithms

In order to verify the time efficiency of the ultrasound image superresolution reconstruction algorithm in this paper, the algorithm in this paper and the other three algorithms will be used to perform superresolution reconstruction on the ultrasound images of traumatic myositis ossificans of the elbow joint and compare them to ultrasound images.

It can be seen from Figure 8 that the time efficiency of ultrasound image reconstruction using the FISTA algorithm is the best among these four methods. This shows that the algorithm in this paper is effective in the reconstruction of ultrasound images.

## 6. Conclusion

With the increase of high-altitude operations and traffic accidents, the incidence of elbow joint dysfunction after trauma is on the rise, and the disability rate is quite high. The patient's elbow joint dysfunction affects the patient's physical and mental health such as life, work, and social interaction. Seeking the treatment of posttraumatic elbow joint dysfunction is the current clinical treatment difficulty. The treatment effect is not uniform, and the effect reports are quite different. In this article, from March 2019 to September 2020, 500 patients with posttraumatic elbow joint dysfunction were treated with personalized surgical treatment, followed by standardized rehabilitation exercises and celecoxib to prevent the occurrence of heterotopic ossification. From the perspective of the application of compressed sensing theory, we have carried out useful discussions on the problems faced by the compressed sensing theory and found solutions. We made a significant improvement to one of the algorithms, while retaining the advantages of compressed sensing for high-resolution and high-contrast signals or image information. It still has good resolution and contrast when the noise is large, which is beneficial to the recovery of ultrasound images. Using FISTA directly to reconstruct medical ultrasound images, the reconstruction results are not ideal. This paper uses the standard image library to establish a simulation model for FISTA training and testing. By adding different intensities of noise to all images in the image library, the influence of noise intensity on the quality of FISTA reconstructed images is analyzed, and it is found that the FISTA model has requirements on the quality of images and training set to be reconstructed. The original ultrasound image is preprocessed, and the clarity of the texture details of the restored ultrasound image is significantly improved, and the image quality meets the requirements. This article uses FISTA as the basic model, and the structure of FISTA is relatively large, which occupies a large part of the memory space. At the same time, a large model will also affect the processing time of the algorithm. Therefore, how to ensure the reconstruction quality of ultrasound images while reducing the network structure is a direction that can continue to be studied.

## Figures and Tables

**Figure 1:** Schematic diagram of specific exercise plan after elbow joint dysfunction release.

**Figure 2:** FISTA algorithm flow.

**Figure 3:** PSNR of ultrasound image reconstruction for different training sets.

**Figure 4:** SSIM reconstruction of ultrasound images with different training sets.

**Figure 5:** Comparison of ultrasound image reconstruction results of traumatic myositis ossificans of the elbow joint. (a) Original image. (b) Bicubic interpolation image. (c) FSRCNN image. (d) US-FSRCNN1 image. (e) FISTA image.

**Figure 6:** PSNR of ultrasound image reconstruction under preprocessing operation.

**Figure 7:** SSIM of ultrasound image reconstruction under preprocessing operation.

**Figure 8:** Comparison of the reconstruction time of the ultrasound image between the algorithm in this paper and other algorithms.

**Table 1:** Optimized FISTA algorithm running time.

Scene range	32 ∗ 32	64 ∗ 64	128 ∗ 128
Estimated iteration step size (s)	0.26	0.31	0.48
30 iterations (s)	0.32	0.39	0.53
60 iterations (s)	0.37	0.43	0.56

## Data Availability

The data used to support the findings of this study are available from the corresponding author upon request.
